The article "ASC Performance Prediction for Medical IoT Communication Networks" was published in 2021. Journal: J Healthc Eng.

# ASC Performance Prediction for Medical IoT Communication Networks

**DOI:** 10.1155/2021/6265520

**Published:** 2021-05-27

**Authors:** Fagen Yin, Pingping Xiao, Zefeng Li

**Affiliations:** ^1^College of Physical Science and Engineering, Yichun University, Yichun 336000, Jiangxi, China; ^2^Institute of Data Science, City University of Macau, Macau 999078, Macau

## Abstract

Wearable devices are gradually entering the medical health field. Medical Internet of Things (IoT) has been widely used in all walks of medical health. With the complexity of medical health application scenarios, the medical IoT communication networks face complex environments. The secure communication issue is very important for medical IoT communication networks. This paper investigates the secrecy performance of medical IoT communication networks. To improve the secrecy performance, we adopt a cooperative communication strategy. We also use the average secrecy capacity (ASC) as a metric, and the expressions are first derived. Then, a secrecy performance intelligent prediction algorithm is proposed. The extensive simulations are used to verify the proposed method. Compared with other methods, the proposed algorithm realizes a better prediction precision.

## 1. Introduction

With explosive growth of medical health applications, the fifth-generation (5G) mobile communication has been widely used in medical Internet of Things (IoT) networks [1, 2]. Different 5G applications [3–5] widely appear in medical IoT communication networks, which can provide quick and convenient user experience and services [6]. However, due to the medical user mobility, the secure communication issue of medical IoT networks is facing many challenges [7].

For medical IoT communication networks, physical layer security is becoming more and more important [8]. With an eavesdropper, the authors [9] investigated the impact of antenna correlation. In [10], the authors developed a code scrambling scheme and analyzed secrecy performance. Considering the physical layer security, Yan et al. [11] studied the resource allocation problem for the cognitive relay networks. In [12], the authors proposed an optimal power allocation to achieve the secure transmission. Considering the cooperative jamming, Lu et al. [13] proposed a secure transmission scheme.

However, analyzing and predicting mobile secrecy performance are very difficult. Recently, machine learning techniques are applied in 5G wireless communications [14, 15]. In pattern classification, classifying the binary data was realized by the support vector machine (SVM) model in [16]. The extreme learning machine (ELM) model was proposed to detect anomaly states in [17]. In [18], the general regression (GR) model predicted the video transmission quality.

The article "ASC Performance Prediction for Medical IoT Communication Networks" was published in 2021. Journal: J Healthc Eng.

To date, no existing studies have considered the secrecy performance prediction of AF relaying medical IoT communication networks. As a consequence, we summarize the main contributions as follows:

1. The secrecy performance is analyzed with AF relaying scheme. Then, we use the average secrecy capacity (ASC) to evaluate secrecy performance and derive the exact expressions.
2. To realize real-time analysis of ASC, we propose an ASC prediction algorithm based on the BP network. ELM, SVM, and GR methods are examined and compared with the proposed method.
3. We verify the derived ASC results under different conditions. Compared with different methods, the proposed algorithm realizes a better prediction precision and a lower time complexity.

## 2. The Medical IoT Communication Network Model

In Figure 1, the medical IoT communication networks have a mobile source (MS), mobile eavesdropper (ME), mobile destination (MD), and mobile relay (MR). *W*_SR_, *W*_RD_, and *W*_RE_ are the relative geometrical gains of MS ⟶ MR, MR ⟶ MD, and MR ⟶ ME links, respectively.

Transmission power is *E*, which is allocated by *K*. 2-Rayleigh distribution can express the channel coefficient *h* [19].

Firstly, MR receives the signal *r*_SR_ as [20]

(1) $$\begin{array}{c} r_{SR}=\sqrt{W_{SR}KE}h_{SR}x+n_{SR}, \end{array}$$

where *n*_SR_ is Gaussian noise.

In the second time slot, AF is used at MR. MD and ME receive the signals *r*_R*ki*_, *k*∈{D, E}, as

(2) $$\begin{array}{c} r_{Rk}=\sqrt{c_{k}E}h_{SR}h_{Rk}x+n_{Rk}. \end{array}$$

The received SNR_*γ*SR*ki*_ is given as

(3) $$\begin{array}{c} \gamma_{SRk}=\frac{\gamma_{SR\gamma Rk}}{1+\bar{\gamma_{SR}}+\gamma_{Rk}}, \end{array}$$

where

(4) $$\begin{array}{c} \gamma_{SR}=W_{SR}K{\left|h_{SR}\right|}^{2}\bar{\gamma }, \end{array}$$

(5) $$\begin{array}{c} \gamma_{Rk}=\left(1-K\right)W_{Rk}{\left|h_{Rk}\right|}^{2}\bar{\gamma }, \end{array}$$

(6) $$\begin{array}{c} \bar{\gamma_{SR}}=W_{SR}K\bar{\gamma }. \end{array}$$

*γ*_SRk_ is hard to calculate exactly. We approximate *γ*_SR*ki*_ as [21]

(7) $$\begin{array}{c} \gamma_{SRAk}=\frac{\gamma_{SR\gamma Rk}}{1+\bar{\gamma_{SR}}+\bar{\gamma_{Rk}}}, \end{array}$$

(8) $$\begin{array}{c} \bar{\gamma_{Rk}}=\left(1-K\right)W_{Rk}\bar{\gamma }. \end{array}$$

With the help of [22], the PDF and CDF of *γ*_SRA*k*_ are as follows:

(9) $$\begin{array}{c} f_{\gamma_{SRAk}}\left(r\right)=\frac{1}{r}G_{0,4}^{4,0}\left[\frac{r}{\chi_{k}}|{1,1,1,1}_{-}\right], \end{array}$$

(10) $$\begin{array}{c} F_{\gamma_{SRAk}}\left(r\right)=G_{1,5}^{4,1}\left[\frac{r}{\chi_{k}}|{1,1,1,1,0}_{1}\right], \end{array}$$

where

(11) $$\begin{array}{c} \chi_{k}=\frac{\bar{\gamma_{SR}}\bar{\gamma_{Rk}}}{1+\bar{\gamma_{SR}}+\bar{\gamma_{Rk}}}. \end{array}$$

The instantaneous secrecy capacity is given as [23]

(12) $$\begin{array}{c} C=\max\left\{\ln\left(1+\gamma_{SRA\;D}\right)-\ln\left(1+\gamma_{SRAE}\right),0\right\}. \end{array}$$

The article "ASC Performance Prediction for Medical IoT Communication Networks" was published in 2021. Journal: J Healthc Eng.

## 3. Average Secrecy Capacity

The ASC is derived as

(13) $$\begin{array}{c} \bar{C}=\int_{0}^{\infty }\int_{0}^{\infty }C\left(\gamma_{SRA\;D},\gamma_{SRAE}\right)f\left(\gamma_{SRA\;D},\gamma_{SRAE}\right)d\gamma_{SRA\;D}d\gamma_{SRAE}=A_{1}+A_{2}-A_{3}. \end{array}$$

*A*_1_ is given as

(14) $$\begin{array}{c} A_{1}=\int_{0}^{\infty }\frac{1}{\gamma_{SRA\;D}}G_{2,2}^{1,2}\left(\gamma_{SRA\;D}|{1,0}_{1,1}\right)G_{0,4}^{4,0}\left[\frac{\gamma_{SRA\;D}}{\chi_{D}}|{1,1,1,1}_{-}\right]G_{1,5}^{4,1}\left[\frac{\gamma_{SRA\;D}}{\chi_{E}}|{1,1,1,1,0}_{1}\right]d\gamma_{SRA\;D}\\ =G_{2,2:0,4:1,5}^{2,1:4,0:4,1}\left[\begin{array}{c} 0,1\\ 0,0 \end{array}|\begin{array}{c} -\\ 1,1,1,1 \end{array}|\begin{array}{c} 1\\ 1,1,1,1,0 \end{array}|\frac{1}{\chi_{D}},\frac{1}{\chi_{E}}\right]. \end{array}$$

We obtain the *A*_2_ as

(15) $$\begin{array}{c} A_{2}=\int_{0}^{\infty }G_{2,2}^{1,2}\left(\gamma_{\text{SRAE}}|{1,0}_{1,1}\right)\frac{1}{\gamma_{\text{SRAE}}}G_{0,4}^{4,0}\left[\frac{\gamma_{\text{SRAE}}}{\chi_{\text{E}}}|{1,1,1,1}_{-}\right]G_{1,5}^{4,1}\left[\frac{\gamma_{\text{SRAE}}}{\chi_{\text{D}}}|{1,1,1,1,0}_{1}\right]d\gamma_{\text{SRAE}}\\ =G_{2,2:0,4:1,5}^{2,1:4,0:4,1}\left[\begin{array}{c} 0,1\\ 0,0 \end{array}|\begin{array}{c} -\\ 1,1,1,1 \end{array}|\begin{array}{c} 1\\ 1,1,1,1,0 \end{array}|\frac{1}{\chi_{\text{E}}},\frac{1}{\chi_{\text{D}}}\right]. \end{array}$$

We obtain the *A*_3_ as

(16) $$\begin{array}{c} A_{3}=\int_{0}^{\infty }\frac{1}{\gamma_{SRAE}}G_{2,2}^{1,2}\left(\gamma_{SRAE}|{1,0}_{1,1}\right)G_{0,4}^{4,0}\left[\frac{\gamma_{SRAE}}{\chi_{E}}|{1,1,1,1}_{-}\right]d\gamma_{SRAE}=G_{2,6}^{6,1}\left[\frac{1}{\chi_{E}}|{1,1,1,1,0,0}_{0,1}\right]. \end{array}$$

Next, we use the derived ASC expressions to set up the data sets and design the BP prediction model.

## 4. Secrecy Performance Prediction Method

### 4.1. Data Sets

*T*_*i*_ =(*X*_*i*_, *y*_*i*_). *X*_*i*_ is given as

(17) $$\begin{array}{c} X_{i}=\left(x_{i1},x_{i2},\ldots ,x_{i5}\right). \end{array}$$

*X*_*i*_ includes 5 indicators, which are *W*_SR_, *W*_RD_, *W*_RE_, *K*, and $\bar{\gamma }$. The ASC performance is the output *y*_*i*_. By using (13), it can obtain the corresponding *y*_*i*_.

### 4.2. Network Structure

Figure 2 shows the BP structure [24].

### 4.3. Metrics

Two metrics are MSE and AE. For *PP* testing data, they are given as

(18) $$\begin{array}{c} \text{MSE}=\frac{\sum_{z=1}^{PP}{\left(d^{z}-y^{z}\right)}^{2}}{PP}, \end{array}$$

(19) $$\begin{array}{c} \text{AE}=\left|d^{z}-y^{z}\right|. \end{array}$$

The article "ASC Performance Prediction for Medical IoT Communication Networks" was published in 2021. Journal: J Healthc Eng.

## 5. Simulation Analysis

Here, *E* = 1, and *μ* = *W*_RD_/*W*_RE_ (in decibels).

For different channels, we evaluate the ASC performance with$\bar{\gamma }$ = 10 dB in Figure 3. The parameters are given in Table 1. The following observations can be made: (1) increasing *μ* improves the ASC performance; (2) the 2-Rayleigh model can obtain the best ASC performance among the three channels.

In Figures 4–13, we consider SVM, ELM, GR, and RBF [25] methods to compare with the BP network.  Table 2 gives the simulation parameters. The MSE and AE of BP are 0.000232889 and 0.04324, which are the lowest MSE and AE in the five methods. This is because BP has the ability to adapt to the time-varying characteristics and enhance the global stability. It has more computing power than other four methods and can be used to solve the rapid optimization problem.

## 6. Conclusion

An AF relaying scheme was used to improve the ASC performance of medical IoT communication networks in this paper. The ASC expressions were derived. Furthermore, we proposed an intelligent prediction algorithm based on the BP network. The simulation results show that (1) as the *u* increases, the system's ASC performance becomes better and (2) compared with SVM, ELM, GR, and RBF methods, the proposed BP algorithm can obtain a better MSE and AE.

## Figures and Tables

**Figure 1:** System model.

**Figure 2:** The BP structure.

**Figure 3:** The ASC performance versus (*u*).

**Figure 4:** Prediction of BP.

**Figure 5:** AE of BP.

**Figure 6:** Prediction of ELM.

**Figure 7:** AE of ELM.

**Figure 8:** Prediction of SVM.

**Figure 9:** AE of SVM.

**Figure 10:** Prediction of GR.

**Figure 11:** AE of GR.

**Figure 12:** Prediction of RBF.

**Figure 13:** AE of RBF.

**Table 1:** Simulation parameters.

Parameter	Value
*m*	1, 2, 3
*K*	0.4
*W*_SR_	5 dB
*W*_RE_	5 dB

**Table 2:** The parameters for five different methods.

Algorithm	BP	ELM	SVM	GR	RBF
Parameter 1	q: 10 r: 10	q: 18000	c: 128	Spread: 0.054	Spread: 18
Parameter 2	*a*_1_: 0.01		g: 0.011		
Parameter 3	*a*_2_: 0.01				

## Data Availability

The data used to support the findings of this study are available from the corresponding author upon reasonable request and with permission of funders.
